The article "Exploratory algorithms to devise multi-epitope subunit vaccine by examining HIV-1 envelope glycoprotein: An immunoinformatics and viroinformatics approach" was retracted in 2025. Reasons: unreliable results or conclusions; concerns about the peer review; concerns about the authorship.

# Exploratory algorithms to devise multi-epitope subunit vaccine by examining HIV-1 envelope glycoprotein: An immunoinformatics and viroinformatics approach

**DOI:** 10.1371/journal.pone.0318523

**Published:** 2025-02-27

**Authors:** Saurav Kumar Mishra, Kanishka Sithira Senathilake, Neeraj Kumar, Chirag N. Patel, Mohammad Borhan Uddin, Taha Alqahtani, Ali Alqahtani, Hanan M. Alharbi, John J. Georrge

**Affiliations:** 1 Department of Bioinformatics, University of North Bengal, Darjeeling, West Bengal, India; 2 Institute of Biochemistry, Molecular Biology and Biotechnology, University of Colombo, Colombo, Sri Lanka; 3 Department of Pharmaceutical Chemistry Bhupal Nobles, College of Pharmacy, Udaipur, Rajasthan, India; 4 Department of Botany, Bioinformatics and Climate Change Impacts Management, School of Science, Gujarat University, Ahmedabad, India; 5 Biotechnology Research Center, Technology Innovation Institute, Abu Dhabi, United Arab Emirates; 6 Computational Biology Research Laboratory, Department of Pharmacy, Faculty of Health and Life Sciences, Daffodil International University, Dhaka, Bangladesh; 7 Department of Pharmacology, College of Pharmacy, King Khalid University, Abha, Saudi Arabia; 8 Department of Pharmaceutical Sciences, College of Pharmacy, Umm Al-Qura University, Makkah, Saudi Arabia; Cholistan University of Veterinary and Animal Sciences, PAKISTAN

## Abstract

Acquired immune deficiency syndrome (AIDS), a widespread pandemic and severe health issue, is triggered by the human immunodeficiency virus (HIV); there is no specific vaccine to cure this infection, and the situation is worsening. Therefore, this research sought to develop a vaccine with multiple epitopes against this infection targeting envelope glycoprotein (vital in host-cell interaction) through the immunoinformatics and viroinformatics approach. We identified one B-cell, eight MHC-I, and four MHC-II epitopes on its immunogen-assisted screening. In addition, these putative epitopes were conjoined concurrently using a specific linker (EAAAK, KK, GPGPG), including an adjuvant and a His-Tag at the N and C terminal, respectively, to augment its immune reaction. The final constructed entity consists of 284 amino acids; immunological evaluation demonstrated that the developed vaccine possesses antigenic features with a value of 0.6222, is non-allergenic, and has prospective physiochemical characteristics. The secondary and tertiary structures were anticipated, and their quality has been evaluated. Further, docking analysis between vaccines with TLR3 shows a strong molecular interaction with a -20.0 kcal/mol binding energy, and the stability was analysed through the MD simulation (100ns). Moreover, the designed vaccine expression and immune response were analysed, and a high vaccine expression level was found (pET28a (+)) and robust immune response followed by codon adaptation index value 0.94, 58.36% GC content, and the generation of IgM +  IgG, cytokines and interleukin. Based on overall investigation, the developed vaccine stimulates a robust immune response. Nevertheless, laboratory analysis is needed to confirm the protective potency of the vaccine.

## 1. Introduction

HIV infection causes acquired immunodeficiency syndrome (AIDS), which continues to pose an epidemic risk to public health around the globe. Based on the World Health Organization (WHO) global case document, The predicted number of HIV-positive people in 2021 is 38.4-40.1 million, with 84.2 million infected since its conception “(https://www.who.int/data/gho/data/themes/hiv-aids)” [1–3]. It belongs to the family of *Retroviridae*, subfamily *Orthoretrovirinae*, and its genome comprises three structural (Env, Gag, and Pol). Also, it has six regulatory proteins (Rev, Nef, Vif, Tat, Vpr, and Vpu), which collectively encode sixteen viral proteins. However, HIV replication requires three enzymes (reverse transcriptase, invertase, and protease) encoded by structural genes to complete the mechanism [4,5]. HIV-1 causes a majority of AIDS; however, HIV-2 is also infectious and the source of the majority of HIV infections worldwide. HIV-1 is the foremost epidemic culprit [6,7]. The primary challenge posed by this pandemic is its inherent variations, which give rise to numerous hereditary subtypes, creating difficulties in therapeutic development. However, the envelope (Env) glycoproteins gp120 and gp41, which drive viral penetration into host cells for replication and transmission, exhibit the most significant variability, and targeting these proteins will be a lead for the therapeutics developments. The transmission of HIV is dependent on the envelope glycoprotein gp120, which is exposed to the virus’s interface and enables HIV entrance into the host cell [8–10]. Moreover, these virulent factor makes it an ideal target for the vaccine candidate development against HIV. In the current scenario, no specific vaccine is available for this viral infection; however, earlier developed vaccines such as AIDSVAX [11], MRKAd5 [12], and RV144 [13] clinical trials have been successful, but they have some major drawbacks such as AIDSVAX; can only neutralise antibody in homologous virus, MRKAd5; will help to trigger only cytotoxic T-cell responses and RV144 is capable of eliciting CD8 + and neutralising antibody responses yet fails to stimulate CD4 + responses; subsequently, it is unwilling to decrease viral load following HIV infection [7]. Furthermore, while highly active antiretroviral therapy (HAART) effectively decreases AIDS-related mortality by 60%, it is incapable of entirely eradicating the virus from people who have been infected [7,14,15]. Consequently, an efficacious vaccine formulation targeting the HIV viral infection is imperative. As we have seen during another pandemic, COVID-19, the advanced computational approach has rapidly been used in the case of viruses for peptide vaccine and therapeutics design, with time-effective, cost-effective, and high accuracy will help reduce the infection [16–20]. Although several research studies specifically on HIV have also been performed using immunoinformatics, *in silico,* advanced bioinformatics approaches, and successfully designed vaccines [7,10,21–24]. Although no data is available on the envelope glycoprotein (gp120) of the multi-epitope peptide vaccine, it can trigger both the cellular and humoral immune response, which can help develop a vaccine to reduce the complete infection in the host. Therefore, this study aims to use rigorous steps of the immunoinformatics approach to explore and find the immunodominant B and T cell epitopes having strong immunological profiles by investigating envelope glycoprotein (gp120) of HIV-1 for construct a safe and efficient subunit vaccine candidate. In this study, the envelope surface glycoprotein, known for its antigenic characteristics, has been utilised as a target for identifying B-cell and T-cell epitopes and validated through different steps for identifying immunodominant potential epitopes. This study developed a vaccine candidate by predicting the highly immunogenic profile epitopes from the gp120. The specified peptides were coupled utilising various linkers, considering diverse adjuvants. To assess the designed vaccine candidate’s effectiveness, molecular interaction with TLR, vaccine stability with the receptor, bacterial expression, and vaccine-assisted immune activity towards the infection were analysed via docking, dynamics, *in silico cloning* and immune activity simulation.

## 2. Materials and methods

### 2.1. Retrieval of the target protein

The target sequence of HIV-1 was collected from NCBI. The target is selected based on the role it plays in viral infection. Further, in subunit vaccine development, the target protein must have an antigenic and non-allergenic nature that can help activate immunity against HIV-1 viral infection. The VaxiJen v2.0 (https://www.ddg-pharmfac.net/vaxijen/VaxiJen/VaxiJen.html) and Allertop 2.0 (https://www.ddg-pharmfac.net/allertop_test/) servers employed to asses the immunological properties of the target, considering its primary sequence [25,26]. The protein sequence has been examined for possible B and T-cell epitopes to fight this viral infection and used as a vaccine candidate. Fig 1 shows the workflow for the complete investigation followed by different steps.

**Fig 1:** Illustration of the anticipated chronology of procedures in this work.

### 2.2. Identification of B-cell epitope

The investigation and identification of epitopes from B cells is an essential stage in vaccine design, given that it enables an understanding of the immunological mechanisms that govern the antibody’s ability to identify an antigen [27]. As a result, two distinct servers have been implemented to anticipate B cell epitopes in the target precisely. First is the IEDB, which detects linear B-cell by integrating the BepiPred 2.0 (http://tools.iedb.org/bcell/) [28], and the second is ABCpred (http://crdd.osdd.net/raghava/abcpred/), which implemented an ANN (artificial neural network), considering and specifying value [29]. Further from the output data, considering both servers, only overlapped epitopes were further used. As mentioned above, the screened epitope was investigated for its antigenic allergenic, including toxicity utilising ToxinPred (http://crdd.osdd.net/raghava/toxinpred/) [25,26,30]. The accuracy of prediction is enhanced by taking advantage of two separate websites that execute two separate algorithms.

### 2.3. Identification of T-cell epitopes and their assessment

Recognising T-cells is crucial in vaccine development as they drive cellular immunity, a key component of vaccine effectiveness. MHC molecules classify T-cell epitopes as class I and II; epitopes demonstrating allele-specific binding to MHC-I and MHC-II were selected to enhance the immune response by activating cytotoxic and helper T-cells [31,32]. TheNetMHCpan-4.1 (https://services.healthtech.dtu.dk/services/NetMHCpan-4.1/) server was employed to assess the MHC-I. It indicates the binding of epitopes using the artificial neural network (ANN) algorithm [33]. Strong connections were assigned a default threshold of 0.5%, weak connections were allocated a threshold of 2%, a prediction epitope of 9 amino acids was selected, and 12 HLA supertype representative alleles were determined [33]. Predicted epitopes with high strong binding were further studied. However, for MHC-II, restricted epitopes, the Tepitool (http://tools.iedb.org/tepitool/), an IEDB-based platform, was employed [28,34]. The 7-allele method was selected using the median consensus percentile rank ≤  20.0, at a default of 15 amino acids long for identifying immunodominant epitopes [35]. Finally, the immunogenic epitopes were selected based on their having antigenic, allergenic, and non-toxic features for vaccine candidates.

### 2.4. Construction of subunit vaccine

Immunodominant B and T-cell (MHCI and MHCII) peptides were linked to create a vaccine construct (selected based on immunological screening) using EAAAK, KK, and GPGPG, respectively [31,36,]. These employed linkers majorly help in various forms such as the EAAAK will help to reduce steric hindrance in epitopes, KK will help to enhance the solubility of the vaccine construct, and the GPGPG linkers will help to prevent aggregation, maintain flexibility, strengthen stability, and facilitate the construction of formulated vaccine. To improve the immunogenic activity, an adjuvant was included to provide an immunomodulatory effect, the PADRE sequence was incorporated to activate T-helper cells, and poly-histidine tags were added to improve solubility and stability, all of which were joined via EAAAK and GPGPG [37]. Further, the constructed sequence was utilised for secondary and tertiary structure assessment.

### 2.5. Immunological and physicochemical assessments

A subunit vaccine candidate must be antigenic and non-allergenic to have a robust immunogenic profile. The antigenic and allergenic profiles were assessed via the VaxiJen v2.0 (https://www.ddg-pharmfac.net/vaxijen/VaxiJen/VaxiJen.html) [25] and Allertop 2.0 (https://www.ddg-pharmfac.net/allertop_test/) [26] servers. Understanding vaccine biological characteristics is critical. The vaccine ought to trigger a successful immune reaction against the infectious organism. The ProtParam (https://web.expasy.org/protparam/) tool evaluated the designed construct’s physical and chemical features, considering the constructed sequence as an input following default parameters [38].

### 2.6. Evaluation of secondary structure

SOMPA(https://npsa-prabi.ibcp.fr/cgi-bin/npsa_automat.pl?page=/NPSA/npsa_sopma.html) server based on homology modelling was utilised to estimate the 2D features vaccine construct [39] to understand its helix, strand, turn, and coil within the constructed sequence. Furthermore, the PSIPRED 4.0 (http://bioinf.cs.ucl.ac.uk/psipred/) server was also employed to compute the secondary structure assessment of the constructed vaccine sequence [31,40].

### 2.7. Structure modelling, refinement, and validation

The 3D model was modelled via the Robetta (https://robetta.bakerlab.org/) server [41], and the promising design model was selected best on the generated multiple models. The selected output model undergoes further improvement via GalaxyWEB (https://galaxy.seoklab.org/cgi-bin/submit.cgi?type=REFINE) tool to enhance three-dimensional structure correctness and quality [42]. Among the improved models, the model had the best quality, considering all parameters were selected. Further, the SAVE v6.0 (https://saves.mbi.ucla.edu/) server was used to examine the enhanced model quality based on the Ramachandran plot, ERRAT, and Verify3D [43] to estimate the correct and incorrect region [44]. ProSA-web (https://prosa.services.came.sbg.ac.at/prosa.php) server was also deployed to systematically and accurately evaluate the modelled structure [45].

### 2.8. Identification of conformational B cell

The Ellipro (http://tools.iedb.org/ellipro/) program, via the IEDB website, identified discontinuous peptides based on the 3D form using default parameters. The vaccine must contain the conformational B cell epitope within the constructed sequence for the proper immune activity response. Therefore, the Ellipro server used the protrusion index to identify cluster atoms based on structure [46].

### 2.9. Disulfide engineering assessment

Disulfide bond extension enhances the durability and linear form structure by introducing disulfide bond formulation into the structure through cysteine mutation at a particular paired site. Based on the model structure, considering all default parameters, the DbD2 (http://cptweb.cpt.wayne.edu/DbD2/) (Craig & Dombkowski, 2013) webserver was employed.

### 2.10. Analysis of structure flexibility

The CABS-Flex 2.0 (https://biocomp.chem.uw.edu.pl/CABSflex2) application analyses the protein’s structural mobility. In the case of subunit peptide vaccines, the designed vaccine structure must be flexible for optimum functioning and molecular recognition [47]. The analysis was accomplished on the CABS-Flex 2.0 utilising model structure as an input in PDB format, employing 50 cycles, an RNG seed of 8954, and a trajectory period of 50 cycles. Furthermore, the values of 1.40, 1.0, and 1.0 have been considered for temperatures, side chain restraint, and C-alpha restraint [48].

### 2.11. Molecular docking with TLR

The interaction analysis is critical in subunit vaccine design because it allows us to determine the relationship between the target receptor and vaccine candidate, ultimately contributing to the immune response. The ClusPro (https://cluspro.org/login.php) tool was employed for docking analysis [49], considering the constructed vaccine and the target receptor as input. Further, the PRODIGY (https://rascar.science.uu.nl/prodigy/) server determined the final selected docked complex’s bound energy [50]. Furthermore, the molecular interaction in the final selected complex was analysed via PDBSum (https://www.ebi.ac.uk/thornton-srv/databases/pdbsum/) [50,51]. Additional molecular dynamic analysis was performed on the selected docked for structural stability.

### 2.12. MD simulation using normal mode analysis

The iMODS (https://imods.iqf.csic.es/) server has been employed to assess the docked complex’s flexibility by investigating the structural changes within the complex [52]. TLR-Vaccine molecular element structural behaviours are determined by normal mode analysis (NMA), which produces a deformation plot, the eigenvalue variability, B-factor importance, correlations map, and dynamic networks framework to understand the molecular compactness better.

### 2.13. Molecular dynamics simulation of vaccine with TLR and MM‑PBSA calculation

The topology files of the complex were created via “Antechamber Python Parser Interface (ACPYPE)” programs and pdb2gmx [53–55]. The complex was then centred in a cubic box, filled with TIP3P water molecules, and neutralised with 24 Chlorine ions, considering a minimum distance of 0.8 nm and was minimised considering the steps of 100 ps [56], via the steepest descent algorithm [16]. The system was equilibrated to mimic the physiological conditions to bring it to 310 K and 1 bar via the NVT and NPT ensemble. Finally, the MD simulation production step was conducted with a simulation time of 100 ns following the time of 2 fs, and the coordinates were saved every 10 ps [56–59]. Furthermore, the “Molecular mechanics -Poisson-Boltzmann surface area (MM-PBSA)” studies were carried out for the energy calculation of vaccine -TLR complex using the MD trajectory and the g_mmpbsa tool. To achieve this, 100 frames of the trajectory were taken out at fixed intervals of 1ns [54,56,59].

### 2.14. Codon optimisation and expression assessment

The developed vaccine underwent codon optimisation for its expression in the vector [16]. VectorBuilder (https://en.vectorbuilder.com/tool/codon-optimization.html) was used for the codon optimisation in *E. coli K12* for optimum expression and efficacy [16,54,]. The codon adaptation index (CAI) and GC composition ratio indicated optimisation quality [17]. Further, the optimised sequence was cloned in a plasmid (pET 28a (+)) utilising SnapGene (https://www.snapgene.com/) software. The pET28a is a well-known cloning vector in vaccine development due to its ability to express highly soluble viral proteins. It also has multiple cloning sites, which will help incorporate the construct, allowing the tags to be included or excluded accordingly. Further, the presence of kanamycin resistance markers offers a more stable culture for the large-scale production of vaccines [60–62]. The researcher also used other plasmids, such as pET30, which contain additional tags (likewise S-tag); however, due to the presence of an ampicillin resistance marker, it will reduce plasmid stability in prolonged cultures [63–65].

### 2.15. Immune simulation profiling of developed vaccine

The C-ImmSim (https://kraken.iac.rm.cnr.it/C-IMMSIM/index.php) has been utilised to comprehend the developed vaccine’s immune-stimulating characteristics and host immune reaction. Further, a complete final construed sequence was subjected as an input for the immune examination. The time steps of parameters were set as reported previously following the recommended vaccination, such as simulation volume, steps and random seed, along with the hots HLA (Human leukocyte antigens) selection to assess its immune-stimulating characteristics [24,66,67].

## 3. Results

### 3.1. Retrieval of the target protein

Envelop glycoprotein (gp120) is a critical component in the viral envelope’s attachment with the host cell by fusing to CD4, which serves as the primary receptor. This virulent factor renders it an ideal selection for vaccine construction. The Envelop glycoprotein (gp120) sequence (Accession ID; NP_579894.2) in FASTA format was retrieved from the NCBI. The immunogen screening resulted in its antigenicity score of 0.4277, and its non-allergenic feature can be further investigated for vaccine development against HIV-1 viral infection. The protein sequence was also investigated to find immunodominant peptides for prospective vaccine development.

### 3.2. Identification of B-cell epitope

The Envelop glycoprotein (gp120) sequence was analysed using two separate servers, IEDB and ABCpred, to determine the presence of antigenic determinants. The BepiPred 2.0 prediction module was utilised in IEDB for this analysis, whereas ABCpred was employed for a more precise and reliable estimation [28]. Using the IEDB server, we predicted 20 subsequent epitopes with different lengths inside the Envelop glycoprotein (gp120) (S1 Table). The graphical representation shows epitopic (yellow-coloured peaks) and non-epitopic regions (green-coloured slopes) in the predicted epitopes within the Envelop glycoprotein (gp120) (S1 Fig). With ABCpred sever 49 B cell epitopes peptide sequences, 16 mer peptides ranked according to their rank and score values was predicted (S2 Table) [29]. Further, the overlapped analysis found that only 3 epitopes are present in both sever which are overlapped in each other; among them, 2 epitopes are non-antigenic, 1 is antigenic, 2 are non-allergenic, and 1 is allergenic, and all 3 are non-toxic in Table 1. Finally, only 1 B cell epitope has favourable immunogenic properties that were further utilised in vaccine development.

**Table 1:** A list of final selected B cell peptides, including their position and immunological properties.

Sl.No	Position	Peptide Sequence	Antigenicity	Allergenicity	Toxicity
1.	436	ESEIFRPGGGDMRDNW	0.1595 (Probable NON-ANTIGEN)	PROBABLE ALLERGEN	Non-Toxin
2.	442	PGGGDMRDNWRSELYK	0.2849 (Probable NON-ANTIGEN)	PROBABLE NON-ALLERGEN	Non-Toxin
3.	464	EPLGVAPTKAKRRVVQ	1.0087 (Probable ANTIGEN)	PROBABLE NON-ALLERGEN	Non-Toxin

### 3.3. Identification of T-cell epitopes and their assessment

Utilising NetMHCpan-4.1, MHC-I peptides of the envelope glycoprotein (gp120) were determined [33] considering its 12 HLA supertype representative alleles and the MHC-II epitope was computed using the Tepitool [34] an IEDB-based resource considering the 7-allele method [28]. Overall, 40 MHC-II and 30 MHC-II peptides have been identified (S3–S4 Table). Further, the antigen, allergen, and toxicity analysis show that out of 32 MHC-I epitopes, 15 are antigenic,17 are non-antigenic, 14 are allergenic,18 are non-allergenic, and all 32 are non-toxic (S3 Table), and in the case of MHC-II (S4 Table) out of 40 epitopes 13 are antigenic,27 are non-antigenic, 19 are allergenic, 21 are non-allergenic, and all 40 are non-toxic. However, the study found that the overlapped MHC-I and MHC-II play a vital role in the subunit vaccine, so out of these identified epitopes, only 8 MHC-I and 4 MHC-II epitopes overlapped and had dominant immune profiles. As described in Table 2, such epitopes are subsequently incorporated into the formulation of vaccines.

**Table 2:** List of selected overlapped peptides from MHC-I and MHC-II with their restricted position, sequence, alleles, and immunological properties.

Sl.No	Position	Epitopes	Alleles	Antigenicity	Allergenicity	Toxicity
**MHC-I Immunodominant epitopes**						
1.	88	KPCVKLTPL	HLA-B0702	1.5232 (Probable ANTIGEN)	PROBABLE NON-ALLERGEN	Non-Toxin
2.	139	KVQKEYAFF	HLA-A2402	0.7720 (Probable ANTIGEN)	PROBABLE NON-ALLERGEN	Non-Toxin
3.	142	KEYAFFYKL	HLA-B4001	0.6017 (Probable ANTIGEN).	PROBABLE NON-ALLERGEN	Non-Toxin
4.	188	YCAPAGFAI	HLA-B3901	1.3004 (Probable ANTIGEN)	PROBABLE NON-ALLERGEN	Non-Toxin
5.	289	VTIGKIGNM	HLA-A2601	1.7087 (Probable ANTIGEN)	PROBABLE NON-ALLERGEN	Non-Toxin
6.	305	SRAKWNNTL	HLA-B3901	0.5984 (Probable ANTIGEN)	PROBABLE NON-ALLERGEN	Non-Toxin
7.	316	IASKLREQF	HLA-B5801	1.0623 (Probable ANTIGEN)	PROBABLE NON-ALLERGEN	Non-Toxin
8.	468	APTKAKRRV	HLA-B0702	0.9750 (Probable ANTIGEN)	PROBABLE NON-ALLERGEN	Non-Toxin
**MHC-II Immunodominant epitopes**						
1.	143	KEYAFFYKLDIIPID	HLA-DRB1 * 07:01 HLA-DRB1 * 15:01 HLA-DRB3 * 01:01 HLA-DRB3 * 02:02 HLA-DRB4 * 01:01	1.2964 (Probable ANTIGEN)	PROBABLE NON-ALLERGEN	Non-Toxin
2.	185	IPIHYCAPAGFAILK	HLA-DRB1 * 07:01	0.5882 (Probable ANTIGEN)	PROBABLE NON-ALLERGEN	Non-Toxin
3.	236	SLAEEEVVIRSVNFT	HLA-DRB1 * 03:01 HLA-DRB1 * 15:01	1.1081 (Probable ANTIGEN)	PROBABLE NON-ALLERGEN	Non-Toxin
4.	464	EPLGVAPTKAKRRVV	HLA-DRB5 * 01:01	1.2335 (Probable ANTIGEN)	PROBABLE NON-ALLERGEN	Non-Toxin

### 3.4. Construction of subunit vaccine

Based on the rigorous steps, only one B-cell, eight MHC-I, and four MHC-II peptides passed all steps, and it was found that these epitopes have the potential immunogenic profile among the predicted epitopes. The B-cells were linked with the MHCI via a KK linker, whereas the eight MHC-I were fused using an EAAAK linker. The MHC-I and MHC-II are attached through the GPGPG, and the 4 are joined with the same linker. Investigation suggests that β-defensin 3 (UniProt ID; Q5U7J2) could improve the function of antigen-presenting cells (APCs) and aid in stimulating innate immunity, which leads to the production of cytokines and chemokines [68] and fusion of the PADRE sequence will aid in activating and initiating innate immune activity. Consequently, β-defensin 3 has been employed at the N side to enhance immunological capabilities and preserve it from degradation. Further, using the EAAAK linker, the β-defensin 3 with B-cell epitope was connected considering the PADRE (AKFVAAWTLKAAA) sequence in between the Adjuvant and B cell, and additionally, the GPGPG linkers tied His-tag at the C-terminal regions [31]. Fig 2 shows the systematic representation of the 284-sequence vaccine construct.

**Fig 2:** A graphical illustration of epitope-based vaccine construction.

### 3.5. Immunological and physicochemical assessments

In an immunological investigation, the vaccine had a beneficial antigen score of 0.6222, demonstrating non-allergenicity. In addition, the physiochemical properties were determined through the Protparam, which are presented in Table 3. The vaccine design’s measured molecular weight (MW) is 30366.62 Da, appropriate for eliciting immune-modulating responses. The peptide’s theoretical pI of 9.95 demonstrates that it is relatively basic. A predicted aliphatic index of 73.10 was obtained, suggesting the protein exhibits thermostable. The protein instability index was computed to 39.08, which is considered stable. The vaccine construct was determined to have a grand average hydropathicity (GRAVY) score of -‒0.315, which represents hydrophilicity and is likely to participate in interactions with water molecules. The various properties corresponding to immunological and physiochemical properties revealed a potent profile (Table 3).

**Table 3:** The computed immunological and physicochemical features of the constructed vaccine.

Sl.No	Properties	Remarks
1.	Antigenicity	0.6222 (Probable ANTIGEN)
2.	Allergenicity	Non-allergenic
3.	Molecular formula	C_1371_H_2205_N_395_O_364_S10
4.	Number of amino acids	284 aa
5.	Molecular weight (MW)	30366.62 Da
6.	Theoretical (pI)	9.95
7.	Half-time estimation	30 h (mammalian reticulocytes, in vitro) >20 h (yeast, in vivo) >10 h (Escherichia coli, in vivo)
8.	Protein instability index (II)	39.08 (Stable)
9.	Aliphatic index	73.10
10.	Grand average of hydropathicity (GRAVY)	–0.315

### 3.6. Evaluation of secondary structure

SOPMA was utilised to examine the two-dimensional structure of the constructed vaccine [39]. The vaccine comprises an alpha helix (55.99%), an irregular coil (32.04%), and an extended strand (11.97%), as determined by the investigation of secondary composition. Fig 3 illustrates the secondary arrangement of the developed candidate, evaluated by utilising the PSIPRED 4.0 software [40,69].

**Fig 3:** A graphic illustration of the secondary structure considering strand, helix, and coil.

### 3.7. Structure modelling, refinement, and validation

The Robetta online program anticipated the vaccine’s tertiary structure [41]. The platform provides five distinct query sequence templates. However, the first model was selected for further examination since 0.48 is the confidence score for each anticipated model, which falls under the acceptable range of confidence score level (from 1.0 to 0.0). After that, the selected model was used as input for refinement through GalaxyRefine [42]. The GalaxyRefine created five optimised vaccine construct models. Within these models, model 4 (Table 4) was selected considering all parameters [70]. Fig 4 illustrates the raw and refined predicted model. Moreover, the engineer’s structure was validated by employing various servers. This was achieved by assessing the enhanced three-dimensional model’s Z-score value, general quality aspect, and Ramachandran chart [43–45]. The enhanced model, as indicated by the four distinct forms, is as follows: the most favoured region (92.8%), the in-addition allowed region (5.5%), the generously allowed region (0.9%), and the restricted region (0.9%) (Fig 5A). The vaccine model’s general quality feature was also determined through the ERRAT and verify 3D (S2 Fig) offering additional proof for its enhanced structure as a superior model (Fig 5B). The improved model’s Z-score was also determined using ProSA online and reported to be ‒6.66, which is consistent with scientifically proven protein structures (Fig 5C). Overall, the vaccine model is good and can be implemented in molecular docking investigations to evaluate target receptor immune reactions.

**Table 4:** List of refined models obtained by GalaxyRefine along with different attributes.

Model	GDT-HA	RMSD	MolProbity	Clash score	Poor rotamers	Rama favored
Initial	1.0000	0.000	1.317	1.5	0.0	93.6
MODEL 1	0.9798	0.304	1.745	8.3	0.5	95.7
MODEL 2	0.9798	0.307	1.673	7.4	0.0	96.1
MODEL 3	0.9736	0.320	1.716	7.2	0.5	95.4
**MODEL 4**	**0.9815**	**0.303**	**1.690**	**7.2**	**0.0**	**95.7**
MODEL 5	0.9736	0.340	1.705	8.1	0.0	96.1

**Fig 4:** An illustration of the tertiary structure of constructed vaccine candidate (A) The constructed initial structure of vaccine candidate (B) Illustration of improved vaccine structure via refinements.

**Fig 5:** The structural validation of the refined vaccine model. (A) Representation of the Ramachandran plot of the designed vaccine construct, and (B) the Z-score representation value of the designed model.

### 3.8. Identification of conformational B cell

Identifying conformational B cells within the vaccine can help understand the immune profile of the developed vaccine as the antibodies recognise it. Thus, employing different parameters, the Ellipro tool at IEDB examined vaccine conformational epitopes [46].

The 5 possible epitopes comprised a total of 139 residues, and values associated with these residues varied from 0.632 to 0.779, and each antigen’s residue count varied from 14 to 48, as shown in S5 Table. Further, all identified conformational B-cell epitope scores were > 0.50, and considered putative B-cell conformational epitopes were shown in Fig 6 (A to E) according to their residue and score as specified in S5 Table [17,70]. The yellow sphere in Fig 6 shows the residue involved as a conformational epitope in the designed vaccine.

**Fig 6:** Illustration of the identified conformational epitopes within the constructed vaccine in which the yellow sphere represents the epitopic region.

### 3.9. Disulfide engineering assessment

The vaccine’s model was disulfide engineered using Disulfide by Design 2 v2.13. The energy value of less than 2.2 kcal/mol was altered through cysteine to form disulfide bonds and stabilise the structures of proteins [71]. The DbD2 server predicted 16 pairings of residues. Only two projected residue pairings had values under 2.2 kcal/mol [72]. Additionally, after assessing the energy measurement values, it was determined that the residues PRO75-LYS79 and CYS89-GLY214 exhibited significant potential for disulfide bond formation. Therefore, these residues were modified by alteration to cysteine residues. The representation of the normal and mutated model (based on the disulfide bonds) is shown in Fig 7 [70].

**Fig 7:** Illustration of the Disulfide bond formulation in the vaccine. (A) The vaccine preliminary 3-D structure; (B) Represents the modified vaccine design (based on disulfide bonds formulation); small yellow rods show bond creation.

### 3.10. Analysis of structure flexibility

Following modelling and refining, the model candidate underwent a structural adaptability evaluation employing the CABS-flex 2.0 server. This evaluation yielded ten alternative models of the applied query model [47]. The RMSF values observed for positions 256 (Higher) and 7 (Lower) have been 6.4630 angstroms and 0.2320 angstroms, respectively. The outcomes demonstrate (Fig 8) that the designed vaccine is suitable and can be employed in further investigations.

**Fig 8:** The structural flexibility analysis of the designed vaccine: (A) An estimated superimposed vaccine models, and (B) The summary of expected root mean square deviation within the designed vaccine model followed by higher and lower fluctuation.

### 3.11. Molecular docking with TLR

Implementing ClusPro 2.0 [49], the molecular interaction procedure was carried out to evaluate vaccine construct interactions with TLR3 receptors (PDB ID: 2A0Z). Following the cluster size and energy score, this generates and ranks thirty docking models (from zero to twenty-nine). Among them, cluster 6 has an inadequate energy score (‒1063.2 kcal/mol), and centre energy (the energy between TLR3 and the designed vaccine) of ‒850.2 kcal/mol was selected (S6 Table). The PRODIGY tools were utilised to project the binding affinities of the identified docking complex, which were ‒20.0 kcal/mol [50]. Additionally, the molecular binding and surface interaction analysis using PDBsum [51] revealed 47 residues of TLR3 interacting with 43 residues of the vaccine construct. 26 hydrogen links, 11 salt bridges, and 252 non-bonded interactions comprise the surface interaction in the vaccine (Chain B) and TLR3 receptors (Chain A). The specific interacting residue between the TLR3 and vaccine and the surface interaction between the complex is depicted in Fig 9.

**Fig 9:** An illustration of molecular interaction activity within the docked complex (TLR3-Vaccine). (A) The surface interaction between vaccine and TLR3, (B) The residue interface interaction between vaccine and TLR3, (C) The different types of interaction between TLR3 (Chain A) and vaccine (Chain B) residues.

### 3.12. MD simulation using normal mode analysis

The ultimate best-docked complex (TLR3 and vaccine component) was examined using NMA-assisted simulation using the iMODS website to assess protein stability [52]. High hinges, which imply high deformation, reflect each residue’s distortion, determining the ability to deform the paired complex (Fig 10A). B-factor values are obtained by applying NMA, a shorthand for protein flexibility derived from atomic movement parameters (Fig 10B). The eigenvalue estimated for the dock complex consists of TLR3 and the vaccine component, and mobility rigidity indicates the energy needed to transform the structure at 1.864628e-05 (Fig 10C) [73]. The complex eigenvalue of each mode of normality has an inverse correlation with its variance (Fig 10D), which is favoured. The distribution of covariance illustrates the reciprocal motion between couples of amino acid segments; correlated, uncorrelated, or anti-correlated connections reflect the various combinations (Fig 10E). The elastic network establishes the linkage connecting between the atoms by measuring their rigidity degree, indicating which combination of atoms is linked by spring and the compactness. The nodes in the graph are colour-coded depending on their rigidity, with more assertive nodes presenting as more significant degrees of grey (Fig 10F). Hence, the various components of the docked complex’s simulation precisely represent the ideal vaccine’s optimum durability.

**Fig 10:** The simulation assessment of docked complex (TLR-3 and vaccine). (A) Deformability of the complex (B) Stability of complex through B-factor using NMA (C) Eigenvalue corresponding to the docking complex (D) The depiction of accumulated and individual variance of the structure (E) Matrix of correlations for the residue index (F) Elastic network model showing connection spring map.

### 3.13. Molecular dynamics simulation of vaccine with TLR and MM‑PBSA calculation

The stability of the complex between the vaccine construct and TLR3 was evaluated in its solvated form for 100 ns using MD simulations (Fig 11) using GROMACS software. During the entire simulation time, RMSD (Fig 11A) variation was less than 1.75 nm, indicating the complex’s stability within the acceptable limits for a vaccine construct [16]. TLR3 receptor showed fewer structural fluctuations relative to the vaccine construct, indicating some flexibility (Fig 11B) during the interaction with TLR3. The vaccine did not dissociate from TLR3 during the simulation period and maintained strong contact with binding energy values ranging from ‒170 kcal/mol to ‒220 kcal/mol (Fig 11C).

**Fig 11:** Representation of stability and interaction energy of the complex between TLR3 and the vaccine. (A) Root mean square deviation (RMSD), (B) root mean square fluctuation (RMSF), (C) binding energy between TLR3 and the vaccine calculated using the MMPBSA method.

### 3.14. Codon optimisation and expression assessment

Using VectorBuilder, the core construct sequence was fully optimised [54]. Moreover, the optimised codon was 855 in length. With a CAI score of 0.94, the optimised GC percentage arrangement increased by 58.36% and fell in the permissible CAI range (0.8–1.0) [17]. These vaccine construct values ensure a high gene expression rate (*E. coli -strain K12*). The SnapGene software was used to clone the modified sequence in the pET28a (+) vector, considering the specific restriction site enzyme was discovered to be 6148 bp (Fig 12). The red colour indicates the location of the incorporated vaccine in the pET28a (+) plasmid.

**Fig 12:** An illustration of the cloned vaccine in the plasmid vector. The red region indicates the vaccine area, and the black region indicates the plasmid vector.

### 3.15. Immune simulation profiling of developed vaccine

The vaccine candidate’s immunological stimulation was assessed via C-ImmSim [66,74] server to understand the potential immunological efficacy, as shown in Fig 13. The simulation-based immune analysis of the proposed vaccine candidate demonstrates that it may induce cellular and humoral defences necessary for eliminating and eradicating HIV-1 viral infection. The antibodies produced after the generation of IgM +  IgG and extended immune responses were seen, followed by IgG1 +  IgG2, IgM, IgG1 and 2, which are beneficial for figuring out how primary, secondary, and tertiary immune reactions emerge (Fig 13A). The Increased concentrations of IFN-γ (2 * 10^6^ ng/ml) and IL-2 (1.4 * 10^6^ ng/ml) approximately exhibit elevated levels of defence mechanisms oriented at combating the HIV-1 viral infection because NK and T cell stimulation is the main trigger of IFN-γ expression. Nonetheless, vigilance was retained until the fifteenth day, as shown in Fig 13B; D is the diversity metric (Lower D values diminish diversity) (Fig 13C). Considering the scale of the immune response (450–500 cells/mm3), the number of functioning B cells per indication appears to be considerable. Activated cytotoxic T cells (Tc) and helper T lymphocytes (Th) increased progressively and persisted in their proliferation throughout the period, as shown in Fig 13D and E.

**Fig 13:** Assessment of vaccine-generated immune response via C-ImmSim. (A)The antibodies produced after the generation of IgM +  IgG, IgM, illustrate the growth of antibodies in response to different levels of antigen (B). Changes in the release of cytokines, notably IFN and IL-2, continued across the fifteen days (C) Productive B cell (purple) release after antigen stimulation of the population per entity-state (D) CD8 lymphocytes that are distinct between entity-states and (E) It exhibits the overall number of T-helper cells in each entity-state adhering to frequent antigen exposure.

## 4. Discussion

As a result of increasing fatality and rates of infection, the spread of HIV has become recognised as an alarming global public health catastrophe. While HIV-1 and HIV-2 have been classified independently, HIV-1 is the most prevalent manifestation of AIDS [1,75]. Several important proteins complete the transmission of the disease in humans. Among them, envelope glycoprotein (gp120) primarily infects the host receptor for viral infection transmission. Therefore, due to its virulence factor, envelope glycoprotein (gp120) could serve as a novel vaccine design candidate [76]. There is no specific treatment available to combat this viral infection; however, earlier-developed vaccines and retroviral therapy have low accuracy, and they are unable to fight this infection [7,11–15]. During the pandemic, epitope-based peptide vaccines emerged as fundamental and effective strategies for combating diseases. While computational biology and immunoinformatics techniques have facilitated the design of peptide vaccines by leveraging immunological data through rigorous validation processes, researchers are increasingly drawn to this approach due to its cost-effectiveness and rapid development timeline [16–19,77,78]. However, multiple investigations have already been performed considering gp120 as a target for different findings, and no data is available for the immunoinformatics and viroinformatics-based, based subunit vaccine design [10,79,80]. Thus, this study used envelop glycoprotein (gp120) to recognise immunodominant B and T-cell epitopes and rigorously evaluate them to develop a highly effective subunit vaccine candidate. Recognition of B and T cell receptors (MHC-I and MHC-II) is vital for evoking immune response in peptide-based vaccine design. B cells release a variety of antibodies against pathogens that lower viral levels, whereas MHC-I (CD8 + T-cell) epitope long-lasting immunity against the infected cell, and MHC-II (CD4 + helper T-cell) can produce both cellular and humoral immune to eradicate viruses and remove contaminated cells from the host [81,82]. Whereas such epitopes possess a capacity to induce action by CD4 + helper T-cells, resulting in the generation of memory cells that can start signalling to activate the B-cell response to neutralisation of the antigens and eliminate viral loads [83,84]. The potential B-cell epitope was identified using two sequential servers selected for their favourable features [28,29] to identify the potent epitope for robust immune response. Subsequently, the T cell epitope was computed through the NetMHCpan-4.1 server and Tepitool server, considering different HLA types for broad population coverage [33,34]. Among the identified epitopes, only overlapped epitopes, i.e., 8 (MHC-I) and 4 (MHC-II), had required features and were selected for subunit vaccine construction [31,36,37]. Among these utilised epitope several epitopes such as KPCVKLTPL [85], KVQKEYAFF [86], KEYAFFYKL [87], YCAPAGFAI [88,89], VTIGKIGNM [90–92], SRAKWNNTL [93,94], APTKAKRRV [95,96], IPIHYCAPAGFAILK [97] are also earlier reported in the HIV infection studies and found to have the potential role. These prior investigations supported this subunit vaccine as a peptide vaccine candidate. The designed vaccine is non-allergenic and antigenic, with a score of 0.6222, which is comparably higher than the earlier reported, i.e., 0.45 [23]. Similarly, the 2D and 3D structure assessment revealed that the designed vaccine has the most promising score in terms of the helix (55.99%), Ramachandran’s favoured region (92.8%), which is comparably higher than the previously reported [23]. In addition, the structural mobility shows that the design is of good quality [47,48]. The molecular interaction in the vaccine and TLR3 was examined to assess its interaction, where it revealed that the vaccine and TLR3 are strongly binding with each other and showing strong binding affinity (20.0 kcal/mol) as well as a higher number of interface interaction residue [73]. Further, the mobility of macromolecules via NMA examination shows that the eigenvalue was 1.864628e-05, which indicated higher adaptability [98]. The simulation additionally showed the constant stability of the docked complex, with just slight fluctuations. The bacterial expression was analysed and cloned in the pET28a (+) vector, and it found that the designed vaccine had a maximum level of expression followed by their GC% (58.36%), which is comparably higher than the previously reported [23]. Moreover, targeting the pET28a (+) in the case of virus-associated infection was found as suitable as in cloning as reported, having the GC% value 51.15 [70], 54.34 [99], 49.74% [100], which lies under the high expression levels of percentage range 30 to 70%. Additionally, the vaccine-generated immune response shows the capability via the generation of (IgG1 +  IgG2), IgM, and other cytokines having high values nearly similar and higher than the previously reported study [18,101], which revealed the capability of the formulated vaccine to induce the immune response. Similar to other studies the immune activity generated towards the response of antigen level within the stipulated time frame of injection was found as suitable to evoke the immune response based on the generated immunoglobulins and many dendritic cells, macrophages, and NK cells as reported [63,102,103] and are capable to reduce the antigen count level. Moreover, in the case of HIV infection, one of the hurdles behind successful vaccines is the low immune response activity of the vaccine. Therefore, in this study, the main found was to screen out the most immunodominant epitope having the immunodominant profile was selected to formulate a vaccine which is precisely based on the B and T cell epitope that targets both cellular and humoral immune and can induce trigger the immune system to reduce infection. The considerable immunodominant characteristics of the constructed subunit vaccine demonstrate that our vaccine formulation is an effective peptide vaccine for fighting HIV-1 viral infection.

## 5. Limitation and future scope

Based on the overall investigation, the formulated vaccine demonstrates promising activity; however, this study has certain limitations. Integrated bioinformatics and viroinformatics approaches were employed in crucial steps, relying on various tools, servers, and databases to design the vaccine candidate. While the vaccine exhibits robust activity, future steps should include experimental validation of the vaccine model, assessment of its efficacy across diverse populations, and evaluation of vaccine-induced immune responses against the infection, followed by different phases of clinical trials.

## 6. Conclusion

HIV is an ongoing pandemic with a high transmission and fatality rate, and no specific vaccine is available to combat this infection. For this investigation, we utilised a sophisticated approach combining immunoinformatics and viroinformatics to develop a subunit vaccine for HIV-1 utilizing immunodominant epitopes derived from the envelope glycoprotein based on immunogen-assisted screening. The vaccine’s interaction with TLR3 was highly stable, as indicated by the results of the molecular interaction and stability investigations. Moreover, the *in silico* cloning in plasmid vector and immune simulation analysis confirmed that the formulated vaccine exhibits an encouraging immunological profile and can elicit an adequate immune response to fight this viral infection. However, additional lab investigations are required to assess the vaccine’s reliability and efficacy.

## Supporting information

S1 Table List of predicted B-cell epitopes along with their start-end position, sequence, and length. (DOCX)

S2 Table List of predicted B-cell epitopes along with the rank, sequence, start position, and corresponding score. (DOCX)

S3 Table List of identified MHC-I epitopes along with their corresponding position, alleles, and immunological properties. (DOCX)

S4 List of identified MHC-II epitopes along with their corresponding position, alleles, and immunological properties. (DOCX)

S5 Table List of predicted conformational B-cell epitopes residue within the vaccine construct. (DOCX)

S6 Table List of the obtained cluster of docked complexes (TLR3-Vaccine) with their representative and their corresponding score; selected complex highlighted in blue color. (DOCX)

S1 Fig Representation of predicted B cell epitopes in the target protein via BepiPred 2.0 Server; yellow represents the epitopic, and green represents the non-epitopic region. (TIFF)

S2 Fig Illustration of 3D structure assessments of vaccine refined model. (A) The representation of the plot assessed via the ERRAT and (B) The representation of the plot assessed via the Verify3D assure the favored feature of the vaccine model.
(TIFF)
